# A Comparison of Decision Tree Algorithms in the Assessment of Biomedical Data

**DOI:** 10.1155/2022/9449497

**Published:** 2022-07-07

**Authors:** Fahima Hajjej, Manal Abdullah Alohali, Malek Badr, Md Adnan Rahman

**Affiliations:** ^1^Department of Information Systems, College of Computer and Information Sciences, Princess Nourah bint Abdulrahman University, P.O. Box 84428, Riyadh 11671, Saudi Arabia; ^2^Department of Medical Instruments Engineering Techniques, Al-Farahidi University, Baghdad 10021, Iraq; ^3^Research Center, The University of Mashreq, Baghdad, Iraq; ^4^Green Business School, Green University of Bangladesh, Bangladesh

## Abstract

By comparing the performance of various tree algorithms, we can determine which one is most useful for analyzing biomedical data. In artificial intelligence, decision trees are a classification model known for their visual aid in making decisions. WEKA software will evaluate biological data from real patients to see how well the decision tree classification algorithm performs. Another goal of this comparison is to assess whether or not decision trees can serve as an effective tool for medical diagnosis in general. In doing so, we will be able to see which algorithms are the most efficient and appropriate to use when delving into this data and arrive at an informed decision.

## 1. Introduction

Over time, many methods for data analysis have been developed, which are mainly based on statistical techniques. However, as the information stored grows considerably, traditional statistical methods have begun to face efficiency and scalability problems. Because most of this information is historical and comes from various sources, it seems clear that there is an imminent need to seek alternative methods for the analysis of this type of data and, from them, to obtain relevant and nonexplicit information. The analysis and interpretation of the data in most cases are made manually; that is, the specialists analyze and prepare a report or a hypothesis about the said data to later reach a conclusion and from this make important decisions and significant. These processes are often very slow and expensive. When the volume of data is excessively large, it exceeds human capacity; then, it becomes very difficult to analyze it without the help of the appropriate tools. Also, with the help of these tools, we can reach an accurate diagnosis [1].

In the case of medicine, it is possible to apply alternative methods due to the large number of conditions involved, the symptoms, and the patients. Ideally, doctors could count on the support of a tool that allows them to analyze the symptomatological data of each of their patients to determine, based on previous cases, the most accurate diagnosis, as well as the optimal treatment to follow, which would represent support and help for the doctor. An alternative tool for the prediction and classification of large amounts of data widely used in artificial intelligence is decision trees.

## 2. Theoretical Framework Decision Trees

Various fields employ decision trees as a prediction model. Its primary goal is inductive learning based on observation and logical reasoning. Prediction systems that use rules to express and categorize a sequence of events that occur sequentially are very much like this [1].

A tree is used to symbolize the inductive learning process's information. Trees can be depicted by nodes, leaves, and branches in a visual representation. Classification begins with a root node representing the attribute from which all other attributes are subtracted. There are questions regarding the property or problem in the internal nodes or their children [1]. One of the problem's class variables is represented by the nodes at the end of the graph, known as leaf nodes. There are two stages in the creation process of a decision tree: induction of the tree and categorization. Initial nodes are constructed from training sets, and each node has a test attribute and a part of training data divided according to the possible values of that test attribute.

Decision trees are in the class of supervised machine learning. Decision trees are frequently used because they are easy to implement, can be interpreted easily, are applied to qualitative, quantitative, continuous, and discrete variables, and give reliable results [2]. Decision trees start from a single root. It is a classification tree that progresses towards decision nodes and terminates in labeled leaves. The structure of a simple decision tree is shown in Figure 1. As shown in Figure 1, decision trees consist of roots, branches, and leaves.

After deciding on a test attribute, the training set is divided into two or more subsets; for each subset, a new node is formed and so on. Objects of more than one class in a node generate an internal node; if the node includes only one class, the class label is assigned to a sheet.

When a new object is created and classed, the tree is traversed from its root node to its leaf node, and from there, the object's membership in a certain class is determined. According to the test attribute present in it, the judgments taken at each internal node determine the tree's path. There are many algorithms to generate decision trees, and some that can be found in the WEKA software are the following:

The CART tree is a regression method used to predict values of continuous variables, but when the assumptions to apply this model are not met, its conclusions can be wrong. CART regression trees are a very easy method of interpreting results. The CARTs use historical data, which are used to build regression trees that allow the classification and prediction of new data; these have the advantage that they can easily manipulate numerical variables; their main characteristics are their robustness to outliers or atypical values. [1, 3]. The REETTree decision tree learning method is very easy and very fast to use. This tree is built using the variance information and is pruned using the error reduction criteria. This decision tree classifies only numerical attributes once; the remaining values are obtained from future instances, dividing these instances into information segments [3].

The RandomTree is a randomly drawn tree from a series of possible trees. In this context and other sources of information, we will take “random” to mean that each tree study tree has an equal chance of being tested. Another way of saying this would be that the distribution of trees is uniform. The RandomTree process is a process that produces a random tree of arbitrary permutations [4].

Singh [1] invented C4.5, an algorithm for creating a decision tree. A new version of Quinlan's ID3 algorithm, known as C4.5, has been developed. We will utilize an open-source Java implementation of the C4.5 algorithm, which is the J48 in the WEKA tool, to produce decision trees that may be used for classification.

The J48 algorithm, widely used in data mining, is a decision tree classifier. The J48 classifier is also known as the C4.5 decision tree. This algorithm classifies the data with a top-down distribution. The final decision tree is reached by dividing the data from the attribute with the highest information gain [3]. The decision tree structure starts with a dataset (training set) partitioned at each node resulting in smaller partitions. In this way, a recursive division strategy is followed. In addition to a dataset, a set of attributes is also transmitted. Objects can be an event, an activity, or attributes which are information about that object. Each tuple in the dataset is associated with a class label, determining whether an object belongs to a particular class. It is tried to reach the highest information gain by using the entropy values at each node. It concludes by starting from the branches created by dividing the data with the highest information gain [4]. The first step in the J48 algorithm is to calculate the information gain [5].

The LMT (logistic model tree) provides a very good description of the data. It consists of a decision tree structure with logistic regression functions on the leaves. As in ordinary decision trees, a test on one of the attributes is associated with each internal node [5–7].

Continuing with the trees that we have the M5P (regression tree) in this decision tree, a standard criterion called M5 is used, which is based on a model tree-type numerical decision tree. It is characterized as follows: build trees using an inductive decision tree algorithm, making routing decisions in nodes taken from the attribute values, and each leaf has an associated class that allows calculating the estimated value of the instance through linear regression [6].

## 3. Review of Literature

Kaur and Wasan's [2] research is an example of a similar research project that we will use to understand our project better. We will conduct a series of comparisons with other works similar to ours to better understand our project. Decision trees are classification models used in artificial intelligence (AI) that have a visual component to their decision-making process, she argues in advance. The decision tree classification approach was tested using two datasets that contained real patient medical data. It is safe to say that these findings align with the symptoms that a breast cancer specialist would look for to make the diagnosis. One database comprised 692 cases observed by a single physician, whereas the other contained 322 cases from 19 specialists. To put it simply, the study is aimed at discovering whether decision trees, as a medical diagnostic tool, are relevant. Another article of Patel and Prajapati [8] describes the decision trees and the ID3 algorithm (induction decision tree) to determine whether or not to apply drugs to patients with cardiovascular diseases. This research empirically demonstrates that it is possible to diagnose the need to administer drugs in patients with symptoms of cardiovascular disease, using the variable blood pressure, cholesterol, blood sugar, allergies to antibiotics, and other allergies, through the use of trees of decision with the algorithm ID3 (induction decision tree) implemented in the Java language [9].

Another article that is very similar to the previous one but uses another type of decision tree is that by Moghimipour and Ebrahimpour [10]. They mention that medical science handles large amounts of information. Advanced machine learning (ML) techniques such as decision trees, support vector machines, and logistic regression can uncover hidden patterns in data. Models developed from these techniques will be very useful for medical science, allowing effective decisions. This article allows us to observe the results obtained about the precision capacity of machine learning techniques, after testing them through a set of data related to cardiovascular diseases provided by the UCI repository. After validating the techniques mentioned with the UCI repository, it is obtained that logistic regression offers the highest levels of precision. It should be noted that support vector machine (SVM) and decision tree (ad) techniques offer acceptable results; however, they are not at the level of the results obtained by logistic regression.

Among other investigations, we have one carried out by Jijo and Abdulazeez [10]; this investigation called “data mining techniques applied to the diagnosis of clinical entities” consists of reducing medical error and improving health processes, which is a priority for all health personnel. In this context, the “clinical decision support systems” (CDSS) arise, a fundamental component in the computerization of the clinical layer. With the evolution of technologies, a large amount of data has been studied and classified through data mining. One of the main advantages of using this in the CDSS has been its ability to generate new knowledge. To this end, through the combination of two mathematical models, it is proposed how it can contribute to the diagnosis of diseases using data mining techniques. To show the models used, arterial hypertension was taken as a case study. The development of the research is governed by the methodology most currently used in the knowledge discovery processes in databases: CRISP-DM 1.0, and is supported by the free distribution tool WEKA 3.6.2, of great prestige among those used for data mining modeling. As a result, data mining techniques obtained various behavior patterns about the risk factors for hypertension.

Citing another work, we have the one by Hassani and Emami [9] dedicated to the theme of “intelligent system for prognosis of survival of kidney transplant patient” based on obtaining a system based on the hybrid knowledge for the prediction of time of survival renal graft survival of patients. This is developed from the edition of a case base obtained as a result of knowledge engineering; using WEKA the learning methods that generate the best results in the forecast of the objective trait that is continuous and represents graft survival time are determined.

Regression tree is a classification model formed by combining logistic regression and decision tree. Logistic regression tree is a decision tree with a regression analysis structure. In this tree structure, logistic regression analysis is performed for each tree branch; then, branches are separated using the C4.5 decision tree. The final stage is the pruning stage of the tree [8]. Hospital mortality from acute myocardial infarction, in short, was based on carrying out an approximation to the methodology of CART-type decision trees (classification and regression trees) developing a model to calculate the probability of hospital death in acute myocardial infarction (AMI). The method is as follows: the minimum basic dataset at hospital discharge (CMBD) of Andalusia, Catalonia, Madrid, and the Basque country for the years 2001 and 2002 is used, which includes cases with AMI as the main diagnosis.

Another project that we considered was one called “determination of the efficiency of the output bracket. Through this training, the model adjusts the weights of the hidden neurons to optimize the output. The advantage of mining over nomograms is that it has cancer treatment therapy based on data mining” [11]. The said project consisted of using data mining instead of nomograms since there is a wide variety of algorithms, which can learn from experience. They are made up of input nodes, hidden nodes, and nodes with the ability to resolve complex nonlinear relationships between variables without making any prior assumptions about those relationships.

This next project was more striking since it is based on a slightly better-known theme: dengue. We have an investigation carried out [12] whose research is on the “classification of dengue hemorrhagic fever using decision trees in the early phase of the disease.” This work focuses on applying the classification technique of regression and classification trees (ARC), to find decision rules that allow classifying a patient with dengue in the various forms of the disease based on clinical and laboratory characteristics. Performance was evaluated based on the method's ability to reduce the overall error rate and correctly classify patients [13].

To classify the data, Navada et al. [14] used her article, “decision trees and Bayesian networks for the investigation of genes linked in Alzheimer's disease,” in which she describes the nested judgments that decision trees reflect. It is possible to classify data using a decision tree employed on the data. The nodes, leaves, and branches of a tree are called its anatomical components. Internal nodes are the queries that are asked regarding a specific attribute of the problem, referred to as “root” or “primary” nodes. There is a node for each answer to the questions. Each node has a branch that leads to a list of possible values for the attribute. One of the problem's class variables is represented by the nodes at the end of the graph, known as leaf nodes.

## 4. Materials and Methods

WEKA's main interface (Figure 2) [15], the Explorer, provides menu selection and form filling options for all procedures. There are six tabs to choose from when you click on the window on the WEKA main screen. WEKA permits several uses of its capabilities on a same screen using its Knowledge Flow feature. A feature called Knowledge Flow allows jobs to be done repeatedly through separate processes even if only one action may be performed at a time on the Explorer screen itself. Operation beneath the Explorer window takes place with complete automation and readiness. It is necessary for the user to initiate these transactions when using Knowledge Flow.

If you have some data and want to make a decision tree out of it, consider the following scenario. There are a few steps that you must do before you can begin working with your data. Then, select a decision tree creation method, build a tree, and analyze the results. Using a different decision tree algorithm and assessment approach, this process can be easily repeated. If you want to switch between your results, evaluate models created on multiple datasets and graphically examine both models and datasets, including the classification errors generated by the models under an explorer menu. The data and information that were used to carry out our research consisted of a database created from audiology tests; to this database, the different methods that the classification trees have were applied to verify the effectiveness of each one of them. These data indicate a diagnosis for each patient and the person's characteristics, such as their age and type of eardrum, if they have presented dizziness. Here, the objective is to determine which attributes serve more to predict the diagnosis obtained [15].

Since the CART decision tree has a recursive bipartite structure, it continues until a new split no longer occurs, and in the next stage, pruning starts from the tip to the root. After each pruning, the most successful decision tree is tried to be determined by using the test data. It is tried to reach the highest information gain by generalizing the binomial distribution at each node using the Gini index values obtained. It is said that it does not perform well if there are interrelated variables.

Other data that was also used was a database containing studies on prostate cancer. Still, algorithms that we can find in the regression trees were applied to that database, which present some difference compared to the classification trees. In this study, the objective is to predict the value of PSA (prostate-specific antigen) based on the values of the other characteristics of the patient [16].

One of the main differences that we can find between these two types of trees is that when the “response variable” or to be clearer when our variable of interest is numerical, we speak of regression trees. In contrast, categorical variables are analyzed using regression tree classification, but in any case, the functioning of these two types of trees is relatively similar.

For this reason, if we want to explain and predict characteristics of observations belonging to the objects of a class whose bases can be explanatory or qualitative variables, we will use classification trees, and on the other hand, for an explanatory and predictive model for a dependent quantitative variable whose bases are quantitative variables similarly, we will use regression trees.

Application.

## 5. Results and Discussion

The observations are as follows:

As shown in Figure 3, the J-48 decision tree algorithm manages to be a practically optimal analysis of the entered data, whose characteristics were modified to present us with a less extensive and understandable tree, reaching a 69.5% classification of the variables.

### 5.1. RandomTree

The random tree starts by choosing a predetermined number of random features at each node. In this algorithm, the branches of the tree are not pruned. Indecision trees, while choosing the most informative feature at each node, are not random in the random tree method. A random tree is a tree in which each tree has an equal chance of being sampled or has a “uniform” distribution. However, each node is considered a randomly generated tree from a set of possible trees of random significance. It also allows the estimation of probabilities for categorical variables [17].

The RandomTree decision tree algorithm, no matter how much work was done on its properties looking for an optimal result and a more simplified tree, only managed to analyze 45% of the data entered.  Figure 4 shows the analysis statistics for the best case.

### 5.2. REPTree

The REPTree decision tree algorithm is not a good algorithm to analyze the data that we are working on. No matter how much we tried to increase the percentage of variables evaluated, the algorithm did not present better results.  Figure 5 shows the analysis statistics for the best case.

### 5.3. DecisionStump

The DecisionStump decision tree algorithm with the data entered and the configuration of the analysis properties only evaluated 47% of the variables. Another disadvantage was that it did not present either a schema of the tree or the tree itself.  Figure 6 shows the analysis statistics for the best case.

### 5.4. SimpleCART

The SimpleCART decision tree algorithm presented almost the same disadvantages as the REPTree algorithm with a low percentage when analyzing the variables and with a single level tree, all this with configurations for a better data sampling.  Figure 7 shows the analysis statistics for the best case.

### 5.5. LMT

The LMT decision tree algorithm turned out to be the most efficient algorithm when interpreting the type of data presented by the study data, presenting a well-summarized tree and with 80% of the variables analyzed.  Figure 8 shows the analysis statistics for the best case.

### 5.6. Regression Trees (Prostate Exam): M5P

The M5P regression tree algorithm turned out to be very efficient when interpreting the attributes and variables that the study database presented, presenting a very well-detailed 7 tree with an approximate frequency of 0.61 of the analyzed variables.  Figure 9 shows the analysis statistics for the best case.

### 5.7. REPTree

The REPTree regression tree algorithm is a good algorithm to analyze the data of this class of databases in which we are working since it presented an optimal performance when analyzing the variables evaluated. It presented an approximate frequency of 0.62 (Figure 10).

## 6. Conclusions

The impact that is desired to obtain with the project in applying decision and regression trees as a tool for the prognosis of medical conditions is to take optimal management of the WEKA software [18].

The classification trees are the most competent for these data, more precisely the logistic model tree or LMT [19] classification tree, which statistically turned out to be the type of tree that presented the most efficient results in its result statistics with an average of 80% correct classifications at the time of executing on the data, whose response or interest variables were the Tymp() variable and the speech() variable, which correspond to the type of eardrum and if the person has problems of speaking [7, 20, 21].

After working on another study which was on the prostate specific antigen which handled quantitative variables, we realize that the regression trees are indicated to analyze this type of data, whose most effective tree was the M5 model tree or the M5P [22–25], whose statistics reached an approximate frequency of 0.62 when analyzing the data, and whose variable of interest was the variables of volume and weight of the prostate (level() and weight()).

## Figures and Tables

**Figure 1:** Decision tree structure.

**Figure 2:** WEKA main screen.

**Figure 3:** Classification trees (audiology exam): J48.

**Figure 4:** Analysis statistics for the best case.

**Figure 5:** Analysis statistics for the best case.

**Figure 6:** Analysis statistics for the best case.

**Figure 7:** Analysis statistics for the best case.

**Figure 8:** Analysis statistics for the best case.

**Figure 9:** Analysis statistics for the best case.

**Figure 10:** Analysis statistics for the best case.

## Data Availability

The data used to support the findings of this study are included within the article.
